RETRACTED

# Evaluation of Water Resource Utilization Efficiency in Provincial Areas of China Based on the Unexpected Output SBM Model

**DOI:** 10.1155/2022/9554730

**Published:** 2022-06-28

**Authors:** Xiaheng Zhang, Zekai Lin

**Affiliations:** ^1^College of Business and Trade, Nanchang Institute of Science and Technology, Nanchang 330108, China; ^2^School of Geography and Tourism, Hanshan Normal University, Chaozhou 521041, China

## Abstract

Based on the SBM model including unexpected output, this paper studies the water resource utilization efficiency of 30 provinces in China from 2003 to 2019. The study found that China's water resource utilization efficiency showed obvious provincial differences. The water resource utilization efficiency of most eastern coastal provinces was relatively high, and that of most central and western inland provinces was not high. There are also significant differences among the three regions of the East, the middle, and the West. The utilization efficiency of water resources in the East is the highest, followed by the middle, and the West is the lowest. The redundancy of input factors, such as labor, capital, and water consumption, is the main reason for the low efficiency of water resource utilization, and the redundancy of wastewater discharge also affects the efficiency of water resource utilization. The clustering results show that the utilization efficiency of water resources in most provinces of China is located in medium efficiency area and low efficiency area, and the efficiency needs to be improved. There are relatively few provinces in high-efficiency areas, highlighting that China's water resource utilization still faces severe challenges.

## 1. Introduction

As an important natural resource, water resources are an important prerequisite for human survival and sustainable development. Due to the rapid development of human economy and society, it not only consumes a lot of water resources but also causes serious water pollution. Coupled with industrial wastewater pollution, it worsens water resources [1]. The resulting water resources crisis has become an important factor restricting economic and social development. At present, many countries in the world are facing the problem of water shortage. It is estimated that, by 2025, nearly 40 countries will be seriously short of water resources, and up to 3 billion people will be seriously short of water [2]. For China, the rapid economic growth after the reform and opening up is accompanied by the shortage of water resources and the deterioration of water ecological environment, which has brought great challenges to the utilization of water resources in China. Nationwide, there is a shortage of water resources in China. In 2018, the total amount of water resources in China was 2796 billion m^3^, and the per capita water resources was 2007.57 m^3^/person. Compared with 3246.640 billion m^3^ and 2354.90 m^3^/person in 2016, the per capita water resources decreased, and the per capita water resources were less than 25% of the world average. At the same time, China has a huge demand for water resources. In 2018, China's total water supply was 611 billion m^3^, which is the same as the total water supply. The utilization of water resources is extensive. For example, the effective utilization coefficient of farmland irrigation water in 2015 was 0.53, which is still far from the world level of 0.7∼0.8. China's total freshwater resources account for 6% of the world's total water resources, and the per capita share of water resources is only 2034 m^3^/person, which is 1/4 of the global per capita level. The water consumption per 10,000 US dollars of GDP is 4749 cubic meters, 9.8 times, and 25 times that of the United States and Japan, respectively, which fully shows that the shortage and inefficient utilization of water resources are particularly prominent in China [3]. From the perspective of regional distribution, China's water resources are in an unbalanced state of regional distribution. In addition, the pollution of water resources in China is becoming more and more serious. From 2009 to 2017, the area of waterlogging removal and the area of soil and water loss control in China continued to rise. The total amount of wastewater discharge continued to rise, peaked in 2015, and improved slightly in 2016 and 2017. From the perspective of regional distribution, China's water resources are in an unbalanced state of regional distribution. For example, the water resources in the north are relatively scarce, while the south is vulnerable to waterlogging. The impact of climate change on inter-regional precipitation has been strengthened, the precipitation in the western region has increased, and the precipitation in the northeast and north China has decreased. It can be seen that there are many water resources problems in China, such as insufficient total amount, unreasonable structure, and unbalanced regional distribution. To this end, the state council issued the opinions on the implementation of the strictest water resources management system in 2012, which clearly stipulates three important red lines: water efficiency, total water consumption, and pollution limitation in water functional areas, especially putting the improvement of water resource utilization efficiency in the first place. The proposal of the 13^th^ five-year plan of the Fifth Plenary Session of the 18^th^ CPC Central Committee in 2015 clearly stipulates that “the strictest water resources management system” must be implemented. In view of this, solving the deterioration of water environment and water ecological imbalance and strengthening the protection and utilization of water resources have become an important problem for the Chinese government. It can be seen that there are many water resources problems in China, such as insufficient total amount, unreasonable structure, unbalanced regional distribution and so on. Agricultural water consumption, industrial water consumption, domestic water consumption, and total ecological water consumption all have a negative impact on water resource utilization efficiency, of which domestic water consumption and industrial water consumption have a greater impact [4]. The water resource utilization efficiency is greatly promoted by natural resource endowment, economic development level, degree of industrialization, and technical progress [5]. Therefore, it needs to analyze the influence factors of them. In view of this, solving the deterioration of water environment and water ecological imbalance and strengthening the protection and utilization of water resources have become an important problem for the Chinese government. In order to effectively solve the contradiction of China's current shortage of water resources, we should use scientific methods to objectively evaluate the current utilization efficiency of China's water resources, understand the shortcomings of water resource utilization, and explore the root causes of low efficiency of water resource utilization, which has important guiding significance for China to build a resource-environment-friendly society.

RETRACTED

## 2. Research Review

Water resource utilization efficiency mostly refers to the maximization of the efficiency of water resources in economy, society, and ecological environment of a country or region in order to promote the efficient and sustainable utilization of water resources under limited water resource supply [6]. The utilization of water resources has always been a hot issue in academic circles, and many scholars at home and abroad have conducted indepth research on this issue. The findings mainly include the following aspects:

### 2.1. Evaluation Index of Water Resource Utilization Efficiency

In the construction of evaluation indicators, there are not only single factor indicators such as water consumption per 10000 yuan of GDP [7] but also all factor indicators through the construction of index system [8, 9]. In terms of specific indicators, there are achievements in constructing indicators from the aspects of per capita water resources, industrial water consumption, domestic water consumption, per capita GDP, degree of opening to the outside world, industrial structure, and technological progress [10]. It also includes agricultural water, industrial water, domestic water, ecological water, employment, and fixed asset investment [11]. In addition, 15 indicators are selected from the five aspects of synthesis, industry, agriculture, life, and ecology to build the evaluation index system of water resource utilization efficiency [12].

RETRACTED

### 2.2. Evaluation Method of Water Resource Utilization Efficiency

With the indepth research on the evaluation of water resource utilization efficiency by scholars at home and abroad, they are widely used in evaluation methods, but most scholars use data envelopment analysis (DEA) [13, 14] and stochastic frontier method (SFA) [15, 16]. A few scholars used DEA and Malmquist Index [17], SBM model [18], extended Markov chain and spatial Markov chain model [19], and Tobit regression model [20]. In addition, some scholars also used the LMDI decomposition method [21], principal component analysis method [22], water resource footprint [23], ratio analysis method [24], ecological function method [25], reference method [26], and other methods to evaluate the utilization efficiency of water resources.

### 2.3. Evaluation Object of Water Resource Utilization Efficiency

In terms of specific evaluation objects, many scholars have carried out more research. In the application field, some scholars evaluated the utilization efficiency of industrial water [27], agricultural water [28], and domestic water [29]. In terms of regional scope, some scholars focus on the national water resource utilization efficiency [30–33], while others study the water resource utilization efficiency of some provinces [34, 35] and also study the water resource utilization efficiency of a single province [36]. At the same time, there are also studies on the utilization efficiency of urban water resources [37, 38].

It can be seen that although domestic and foreign scholars have used a variety of methods to evaluate the efficiency of water resource utilization from different angles, the relevant research is still less related to the “unexpected” output generated in the process of water resource utilization, and the used data are relatively old, resulting that existing research results cannot timely and truly reflect the utilization level of water resources. Therefore, this paper constructs an SBM model including “unexpected” output to evaluate the water resource utilization efficiency of various provinces in China and carries out a comprehensive evaluation on this basis, so as to provide an important reference for effectively improving the sustainable utilization level of water resources.

RETRACTED

## 3. Research Method

### 3.1. Nonradial and Nonangular SBM Model

Data envelopment analysis (DEA) is a systematic analysis method developed by operational research scientists, Charnes and Cooper, on the basis of the concept of “relative efficiency evaluation” [39, 40]. DEA is a method to measure the relative efficiency of decision-making unit based on multi-input and multioutput [41]. Compared with the SFA method, the DEA method has incomparable flexibility in dealing with multiple input and output indicators, so it is widely used to evaluate the efficiency evaluation of multiple departments or fields. The principle of this method uses the idea of mathematical programming. Through the predetermined decision-making unit (DUM), on the premise of constant input and output indicators, the mathematical programming method is used to find the optimal frontier and then compare the distance between different decision-making units and the frontier, so as to evaluate the relative effectiveness of different decision-making units. Traditional radial DEA model has not considered the influence of “relaxation variable” on the efficiency value. Moreover, it has not considered the technical changes that increase the expected output and reduce the unexpected output at the same time. This is not accurate enough to measure the efficiency value. When evaluating the efficiency of water resource utilization, the traditional DEA method only takes into account the single output index of GDP and fails to involve the problem of water pollution in the process of water resource utilization, which is obviously inconsistent with the actual situation of water resource utilization. In addition, the relaxation problem caused by the input index and output index cannot be analyzed, which leads to the inevitable large error of the traditional DEA method in calculating the efficiency of water resource utilization. Based on this, in order to solve this problem, Tone proposed an environmental efficiency evaluation model based on input and output relaxation variables, namely, SBM model in 2001 [42]. On this basis, Tone put forward the SBM extension model in 2004, so as to realize the evaluation of environmental efficiency under the condition of unexpected output [43]. The nonradial and nonangular SBM model proposed by Tone, which includes unexpected output indicators, has the greatest feature that it can accurately calculate the relaxation value of input-output indicators in the process of measuring efficiency, which is helpful to improve from ineffective efficiency to effective efficiency.

RETRACTED

Compared with the traditional DEA model, the SBM model calculates the relaxation variable of the input-output index to the greatest extent, so as to measure the efficiency value of the investigated object. It is assumed to build a complete production system, which includes N decision-making units (DMUs). Each decision-making unit needs to input *m* units of production factors in the operation process, so as to produce S_1_ units of expected output and S_2_ units of unexpected output.

Assuming that the final decision-making unit is expressed in *DMU*_0_=(*x*_0_, *y*_0_^*g*^, *y*_0_^*b*^) and the element input variable is *X*=(*x*_1_, *x*_2_,…, *x*_*n*_) ∈ *R*_+_^*m*×*n*^ > 0, the expected output and unexpected source are expressed as follows:

(1) $$\begin{array}{c} Y^{g}=\left(y_{1}^{g},y_{2}^{g},\cdots ,y_{n}^{g}\right)\in R_{+}^{s_{1}\times n}>0, \end{array}$$

(2) $$\begin{array}{c} Y^{b}=\left(y_{1}^{b},y_{2}^{b},\cdots ,y_{n}^{b}\right)\in R_{+}^{s_{2}\times n}>0. \end{array}$$

By setting these assumptions, we can establish the SBM type including the unexpected output:

(3) $$\begin{array}{c} P^{t}\left(x\right)=\left\{\left(x_{0},y_{0}^{g},y_{0}^{b}\right)|x\geq X\lambda ,y_{0}^{g}\geq y_{0}^{g}\lambda ,y_{0}^{b}=y_{0}^{b}\lambda ,\sum_{i=1}^{n=1}\lambda =1,\lambda \geq 0\right\}. \end{array}$$

It can be seen from equation (3) that the equation part of the whole model shows the important characteristics of zero combination of the expected output and unexpected output and joint weak disposability. The inequality part of the model is a constraint condition, which reflects the strong disposability between input variables and output variables. This means that the model is convex and bounded and is used to examine the weight of the cross section of the whole model, *λ*, showing a positive value.

When dealing with these characteristics, the whole operation process of the SBM model is expressed as follows:

(4) $$\begin{array}{c} \min\rho =\frac{1-\left(1/m\right)\sum_{i=1}^{m}s_{i}^{x-}/x_{io}}{1+\left(1/\left(s_{d}+s_{u}\right)\right)\left(\sum_{d=1}^{d}s_{d}^{y+}/y_{do}+\sum_{u=1}^{u}s_{u}^{b-}/b_{uo}\right)},\\ \text{s.t.}\begin{array}{c} x_{o}=\sum_{j-1}^{n}\lambda_{j}x_{ij}+s_{i}^{x-},\;i=1,2,\ldots m,\\ y_{o}=\sum_{j-1}^{n}\lambda_{j}y_{dj}-s_{d}^{y+},\;d=1,2,\ldots d,\\ b_{o}=\sum_{j-1}^{n}\lambda_{j}b_{uj}+s_{u}^{b-},\;u=1,2,\ldots u,\\ \lambda \geq 0,s_{i}^{x-}\geq 0,s_{d}^{y+}\geq 0,s_{u}^{b-}\geq 0. \end{array} \end{array}$$

In equation (4), *s*^*x*−^ ∈ *R*^*m*^, *s*^*y*+^ ∈ *R*^*d*^, and *s*^*b*−^ ∈ *R*^*u*^ represent the relaxation variables of input index, expected output index, and unexpected output index, respectively. If these relaxation variables are greater than zero, it means that there are problems such as input redundancy, insufficient expected output, and undesired output redundancy in the whole model. Equation *ρ* is expressed in the form of ratio. If it is not 1, the molecule represents the proportion that the input index can be reduced in the improvement process of realizing the optimization of efficiency, that is, the input is inefficient. The denominator means that, in the process of efficiency optimization, the expected output can increase or the unexpected output can decrease, that is, the output is inefficient. In the whole decision-making unit, only when the conditions of *s*^*x*−^=0, *s*^*y*+^=0, and *s*^*b*−^=0 are met, that is *ρ*=1, the whole efficiency is optimized. If *ρ* < 1 occurs, it reflects the invalid situation of the whole solution unit. Only by reducing the slack variables of input and output indicators can we ensure that the invalid state of the whole decision-making unit is optimized to an effective state.

RETRACTED

### 3.2. Cluster Analysis Method

Cluster analysis method is used to analyze the regional characteristics of water resource utilization efficiency in China. By setting different grouping criteria, the clustering method divides the water resource utilization efficiency into different groups according to the value of the investigated object. Clustering methods are mainly divided into two different clustering analysis methods: C-means cluster and K-means cluster. Compared with the two, the application of the latter is more flexible and universal. Therefore, the K-means cluster method is selected. The basic principle of the K-means cluster is to assume that the overall sample set is {*x*^(1)^, ⋯, *x*^(*n*)^}, and each sample is *x*^(*i*)^ ∈ *R*^*n*^, *μ*_1_, *μ*_2_,…, *μ*_*k*_ ∈ *R*^*n*^ represented by K-cluster centroids selected to represent the whole sample. K-means cluster is to minimize the distance between the sample and the cluster centroid.

(5) $$\begin{array}{c} J={\sum_{n=1}^{N}\sum_{k=1}^{K}\Gamma nk\left\|x_{n}-\mu_{k}\right\|}^{2}. \end{array}$$

In equation (5), Γ*nk* represents the value range of cluster K. When Γ*nk* is 1, it means Γ*nk* is within the range of cluster K. When Γ*nk* is 0, it means Γ*nk* is outside the scope of cluster K.

Generally speaking, it is very difficult to select the optimal clustering centroid directly by the observation method, which can only be gradually selected by using professional software according to the iterative method. The specific steps are as follows: firstly, assuming that *μ*_*k*_ does not change, it is easier to select the optimal one. On the premise that the whole data point is closest to its central point, the whole function can be minimized. Secondly, assuming that the whole of Γ*nk* is constant, the optimal *μ*_*k*_ is selected. Finally, take the derivative of *μ*_*k*_ and assume that the derivative is zero, then the minimum *J* distance can be calculated finally. Then, the optimal *μ*_*k*_ can be expressed as follows:

(6) $$\begin{array}{c} \mu_{k}=\frac{\sum {}_{n}\Gamma nkx_{n}}{\sum {}_{n}\Gamma nk}. \end{array}$$

In equation (6), *μ*_*k*_ is the average value of data points in the whole cluster K, that is, the optimization is realized. This means that, in each iteration, the value of j-distance is the smallest, so that the whole j-distance will only continue to shrink without increasing and finally achieve a minimum value of K-means. On the premise of obtaining the minimum value, through multiple iterative aggregation, the whole investigation object will be divided into different clustering groups according to the clustering standard.

RETRACTED

### 3.3. Evaluation Index System

Water resource utilization efficiency is a process that includes the ecological value function of water resources, can produce the maximum green economic benefits with the minimum investment of water resources, and ensure the minimization of pollution discharge [44]. In the process of participating in economic activities, water resources can produce not only expected outputs such as GDP but also unexpected outputs such as sewage discharge. In view of this, in order to deeply investigate the utilization and ecological value of water resources, it is necessary to bring unexpected output into the research framework of water resource utilization efficiency.

As an important natural resource, water resources cannot be used alone to measure its utilization efficiency. It must be combined with other production factors to complete the whole economic production activities. In the construction of the evaluation index system of water resource utilization efficiency, the input indexes include the following: first, the participation of water resource consumption as the primary input element not only reflects the degree of water use in a region but also is the key condition to measure the efficiency of water resource utilization; second, as an input factor in economic production activities, labor force is the user of water resource utilization, and it is an essential input factor index in the analysis of water resource utilization efficiency; third, in addition to the necessary natural resources and labor force, capital investment is also an essential factor in the economic activities of a region. Without the participation of capital, the whole economic production activities cannot be completed. Therefore, this paper takes the capital stock as an important input factor index.

RETRACTED

The utilization efficiency of water resources specifically refers to the degree of economic benefits it produces. Therefore, the important output index is the gross domestic product (GDP), which is also the expected output index of the evaluation index system. Because the water resource utilization efficiency includes the ecological and environmental value of water resources, the pollutant discharge generated in the process of water resource utilization is another important output. Therefore, it is necessary to take the wastewater discharge as the unexpected output index of the evaluation index system.

To sum up, the input indicators determined by the evaluation index system of water resource utilization efficiency are water resource consumption, labor force, and capital stock, and the output indicators are divided into expected output indicators and unexpected output indicators, in which the former is GDP and the latter is wastewater discharge.

## 4. Result Analysis

### 4.1. Comparison of Regional Differences in Water Resource Utilization Efficiency

From formulas (3) and (4), the data of input and output indicators are brought into the mSBM model, and the water resource utilization efficiency of 30 provinces and cities in China from 2003 to 2019 is calculated by using MaxDEA software, as shown in Figure 1. From the average value of water resource utilization efficiency of each province, only the water resource utilization efficiency of Tianjin and Shanghai municipalities directly under the central government has been 1 in the sample period, that is, it has reached the frontier of efficiency. The utilization efficiency of water resources in other provinces has not been optimized, and there is some room for improvement.

From the comparison of the differences among various provinces, Tianjin, Shanghai, Shandong, Heilongjiang, and Liaoning ranked among the top five provinces in China in terms of water resource utilization efficiency, and the average value of water resource utilization efficiency exceeded 0.88. Among the five provinces, Heilongjiang is located in the central region, and the other four provinces are located in the eastern region. There are reasons why these five provinces are in the leading position in the country. Tianjin, Shanghai, Shandong, and Liaoning are located in the eastern coastal areas. They are also economically developed areas in China. Their market economy has developed relatively well, their industrial structure has gradually realized the transformation and development from heavy industry to modern service industry, the level of resource utilization intensification has been continuously improved, and water-saving technologies have been continuously innovated, popularized, and applied, resulting in high water resource utilization efficiency. Heilongjiang is a traditional “northern wasteland” area in China. In recent years, the state has vigorously advocated the policy of returning farmland to forests. Heilongjiang's forests and wetlands have been well protected, and the water resources conservation benefits of forests and wetlands rank among the top in the country. The government implements strict water resource utilization policies, so Heilongjiang's water resource utilization efficiency is also high.

RETRACTED

Xinjiang, Guangxi, Guizhou, Qinghai, and Ningxia are the last five provinces in China in terms of water resource utilization efficiency, and their water resource utilization efficiency is less than 0.35. The economic development level is relatively backward, the market mechanism is not perfect, the industrial structure is dominated by traditional agriculture and industry, and the water resource utilization mode is relatively extensive, which are important incentives for the low efficiency of water resource utilization in these provinces.

It can be seen that China's water resource utilization efficiency has significant provincial differences. Most of the provinces with high water resource efficiency are located in the eastern coastal areas; while most of the inland provinces in the central and western regions have relatively low water resource efficiency. Therefore, for China, accelerating the improvement of inland provinces in central and Western China with low water resources efficiency is of great significance to realize the sustainable utilization of water resources.

Analyze the change trend of water resource utilization efficiency according to the eastern, central, and western regions, as shown in Figure 2. On the whole, the national water resource utilization efficiency has little change from 2003 to 2019, and its change trend is relatively gentle. The utilization efficiency of water resources in the eastern region shows an inverted “U” trend in this annual cycle, and its significant change characteristics are “high in the middle and low at both ends.” The change trend of water resource utilization efficiency in the central region is similar to that in the whole country, with little change during the sample period. The only significant change is the significant decline of water resource utilization efficiency in 2017. Taking 2006 as the node, the western region showed a slow decline before 2006, and there was no obvious change after 2006. From the difference of water resource utilization efficiency in each region, the regional differentiation is more obvious. During the period from 2003 to 2019, the average value of water resource utilization efficiency in the eastern region is as high as 0.734, far higher than the national average level of 0.543, the average value of water resource utilization efficiency in the central region is 0.518, close to the national average level, and the average value of water resource utilization efficiency in the western region is only 0.351, far lower than the national average level. It can be seen that the utilization efficiency of water resources in the East is the highest, followed by the middle and the West. The utilization efficiency of water resources shows a decreasing trend from the eastern region to the central and western regions.

RETRACTED

### 4.2. Ineffectiveness Analysis of Water Resource Utilization Efficiency

According to the operation results of the mSBM model, further differential variable analysis is carried out to find out the input factor redundancy, expected output insufficiency, and unexpected output redundancy of water resource utilization efficiency, and then dig out the specific reasons for the ineffective water resource utilization efficiency. On this basis, through the corresponding improvement range, the noneffective DEA decision-making unit is improved into an effective DEA decision-making unit. The input redundancy, expected output deficiency, and unexpected output redundancy of the five provinces with the lowest water resource utilization efficiency in China in 2003 and 2019 are calculated. It can be seen from Table 1 that whether in 2003 or 2019, the main factors leading to the ineffectiveness of water resource utilization efficiency in Xinjiang, Guangxi, Qinghai, Guizhou, and Ningxia are due to the redundancy of labor, capital, and water resource consumption, and the redundancy of total wastewater discharge also has a certain impact.

### 4.3. Regional Cluster Analysis

Based on equation (5) and equation (6), SPSS22.0 software is used for K-means cluster analysis of water resource utilization efficiency of each province. According to the three criteria of high-efficiency area, medium efficiency area, and low efficiency area, the regional case standard is selected, and the clustering results of water resource utilization efficiency of each province are obtained by means of step-by-step iteration and classification. Tianjin, Shanghai, Shandong, Heilongjiang, Liaoning, and Guangdong are in the high-efficiency area of water resource utilization efficiency. A total of 11 provinces, including Fujian, Zhejiang, Jiangsu, Beijing, Hebei, Hubei, Inner Mongolia, Sichuan, Hunan, Anhui, and Henan, are in the medium efficiency zone. Jilin, Jiangxi, Chongqing, Shanxi, Hainan, Shaanxi, Yunnan, Gansu, Xinjiang, Guangxi, Guizhou, Qinghai, and Ningxia are in low efficiency areas. It can be seen that there are relatively few provinces with high water resource utilization efficiency in China, and the number of high efficiency provinces is accounting for only 20%. Most provinces are located in the low campus of the medium efficiency area where the efficiency needs to be improved, and the number of low efficiency provinces is accounting for as much as 80%. The provinces in low efficiency areas are mainly distributed in the inland areas of the central and western regions, which are also the areas that the state should focus on while formulating water resource utilization policies.

RETRACTED

## 5. Conclusion and Discussion

By constructing the SBM model including unexpected output, and on the basis of constructing the evaluation index system of water resource utilization efficiency, MaxDEA software is used to measure the water resource utilization efficiency of 30 provinces in China from 2003 to 2019, and a comprehensive evaluation is carried out accordingly. The results show that (1) the top five provinces in China are Tianjin, Shanghai, Shandong, Heilongjiang, and Liaoning. Except that Heilongjiang is located in the central region, the other provinces are located in the eastern coastal region. The last five provinces in China are Xinjiang, Guangxi, Guizhou, Qinghai, and Ningxia, which are located in the inland regions of the central and western regions. (2) From the perspective of the three major regions of the East, the middle, and the West, the regional differentiation is more obvious. In order, the utilization efficiency of water resources in the East is the highest, the middle is the second, and the West is the lowest. (3) From the perspective of causes, the key factor leading to the low efficiency of water resource utilization is the redundancy of input factors such as labor, capital, and water resource consumption, and the redundancy of wastewater discharge also has a certain impact. (4) The clustering results show that up to 80% of the provinces' water resource utilization efficiency is located in the medium efficiency area and low efficiency area, and its efficiency needs to be improved, and only 20% of the provinces are in the ideal high-efficiency area.

China is still the largest developing country in the world. Although the speed of economic development is still in the forefront of the world, the problems brought by economic growth, including the utilization of water resources are becoming more and more serious, which undoubtedly brings great challenges to China's promotion of sustainable development strategy. China is still facing a dilemma in the utilization of water resources: (1) the rapid development of economy will inevitably lead to a significant increase in the use of water resources, but the utilization of water resources in most provinces is still characterized by certain extensive characteristics. Not only the water-saving technology is lagging behind but also some local governments fail to really realize the importance of efficient utilization of water resources; (2) China's economic development is in a critical period of transformation, and the efficient and economical utilization of water resources, including water resources, has become an important measurement index. However, to truly realize this index, local governments still have a lot of work to strengthen.

RETRACTED

## Figures and Tables

**Figure 1:** Average value of water resource utilization efficiency of various provinces in China during 2003–2019.

**Figure 2:** Change trend of water resource utilization efficiency in China and its three regions.

**Table 1:** Input redundancy, expected output deficiency, and unexpected output redundancy of five provinces in 2003 and 2019.

Province	2003					2019				
	Labor	Capital stock	Water consumption	GDP	Wastewater discharge	Labor	Capital stock	Water consumption	GDP	Wastewater discharge
Xinjiang	−325.023	−228.517	−464.148	0	−1.117	−837.522	−14218.633	−538.418	0	−2.515
Guangxi	−1757.351	−446.254	−227.622	0	−7.292	−2087.719	−22165.515	−233.520	0	−7.121
Qinghai	−171.231	−268.153	−24.472	0	−0.524	−221.819	−4958.217	−23.311	0	−1.522
Guizhou	−1741.457	−404.127	−71.105	0	−3.157	−1577.152	−5322.521	−88.204	0	−5.813
Ningxia	−168.362	−361.468	−79.034	0	−0.329	−278.149	−8071.422	−57.348	0	−1.785

## Data Availability

No data were used to support this study.
